# Research on Students' Satisfaction of Intelligent Learning Based on Text Mining Technology

**DOI:** 10.1155/2022/4024263

**Published:** 2022-06-22

**Authors:** Wei Liu, Yanqiu Zhang, Tongtong Wang

**Affiliations:** Business College of Beijing Union University, Beijing 100025, China

## Abstract

Recently, professionals have highlighted the need for students to have information technology and data analytic skills to be successful in the profession. To meet this demand, educators attempt to integrate technology into curricula. However, the satisfaction of students is of greater importance to evaluating curriculum quality than teaching. This study explores the perceptions that second-year undergraduate students (*n* = 51) enrolled in a Chinese University held about the teaching contents and teaching approaches of intelligent curriculum. Based on the data sample of the students' summary text for curriculum learning, this study adopts TFIDF analysis, topic modeling, text sentiment analysis, and other text mining technologies so as to have a profound analysis on the students' satisfaction. We find that: (1) the students have a higher satisfaction on the teaching contents involved in the financial sharing center compared to RPA financial robot; (2) students have a better adjustment to case analysis and flipped classroom compared to simulation training and classroom lecturing. Our findings and discussion should be of interest to leaders and teachers of business program seeking to integrate technology. We believe that this study's results provide opportunities to have a further improvement of the teaching contents and optimization of teaching design to effectively improve the curriculum quality in order to achieve enhancement of students' satisfaction.

## 1. Introduction

The application of a new generation of information technology, including Internet, big data, artificial intelligence, robot process automation technology, and block-chain, is proceeding with a new round of technical reform and industrial revolution in the world. In the Top Ten IT Information Technologies Affecting Chinese Accounting Practitioners in 2020 held by Shanghai National Accounting Institute in China, financial cloud, e-invoice, big data technology for accounting, e-file, RPA (robot process automation), new-generation ERP, block-chain technology, mobile payment, data mining, and online audit has been enlisted to point a clear direction of the cultivation of accounting talents' core competence. While accountants use of information technology is increasing, their knowledge and understanding still lag behind the broader business community e.g., [1, 2]. As such, enhancing the application of technology and data analytic skills in accounting profession is the focus of discussion for public accounting firms (e.g., [3, 4], the accounting profession at large, e.g., [5, 6], the American Accounting Association (AAA), academics [7–9]. There would be intelligent financial accountants, intelligent financial engineers, intelligent financial operator, and intelligent financial planner for these four posts in the future [10]. The cultivation of compound accounting talents based on intelligent technology has been a consensus for the academic circle and business circle, but there is a serious imbalance between supply and demand [11]. Some Chinese universities have set the major or professional class of intelligent accounting (finance), and such technical curriculums as computer science, intelligent accounting (finance), and big data analysis are added in the compulsory curriculums of traditional accounting [12].

However, we observe a decline in article production of all types in 2019 and 2020 with 81 articles in 2019 and 88 articles in 2020 by consulting five accounting education journals: (1) Journal of Accounting Education, (2) Accounting Education, (3) Advances in Accounting Education: Teaching and Curriculum Innovations, (4) Issues in Accounting Education, and (5) The Accounting Educators' Journal. These total numbers are the lowest since 2006 [13]. The observed declination in the volume of literature addresses accounting education is in severe contrast to the importance of the topic. The COVID-19 crisis undoubtedly exacerbated the impact in 2020 and it becomes extraordinarily difficult to maintain regular teaching and research. Actually, the trend started before the pandemic altered the manner teachers engaging with their students. The review of articles' topics concerned with student issues in accounting education includes CPA exam, value of student organizations to career success, ethical attitudes, student compassion, and learning strategies [14]. These articles reveal a continued interest in empirical examination which make up above 80%. In the context of the pandemic, few studies have examined student satisfaction with the content and style of instruction in courses. Especially, there is a particular lack of research into integrating intelligent technologies into current accounting curriculum content. Our research focuses on undergraduate students' satisfaction with the study of intelligent accounting courses, which is mainly measured from two aspects: teaching content and teaching method.

This paper reports that data are gained from the learning summary and understanding of sophomores after having Intelligent Accounting four times in a business college. A total of 51 students majored in international business, finance, and accounting, including 16 boys and 36 girls took the curriculum. They had submitted 202 texts during the course of study. The main contents include students' evaluation and reflection of the learning contents and teaching methods related to the curriculum. Through a review of literature and introduction of Intelligent accounting curriculum, this study identifies TFIDF analysis, topic modeling, and text sentiment analysis that help create a scientific method. The following sections provide analysis of satisfaction of teaching contents and teaching method based on text mining approaches and systematic process. Followed by the interesting result, we discuss and propose some suggestions and identify potential research opportunities and potential limitations of this research.

## 2. Literature Review

Examining the existing literature's view on intelligent accounting, we will divide this chapter into two subsections. The first section presents relevant research in China. The second section deals with the important papers in other countries.

### 2.1. Relevant Research in China

Under the background of ceaseless integration of big data, artificial intelligence, and accounting, study of accounting education in universities has been a highlight. Wang and Su [15] suggest that artificial intelligence technology is a reformer for accountancy, reporting, and education model of accounting. Therefore, the accounting talents under the background of big data would form a new cultivation mode [16]. Ying and Yang [17] innovatively suggested the artificial accounting mode and the reconstruction of the accounting career. Recently, Renmin University of China, Zhejiang University, and Shandong University have specifically introduced their own cultivation scheme and curriculum system for intelligent financial talents [12, 18, 19]. Cheng and Peng [20] took the MPAcc (Master of Professional Accounting) education of Chongqing University of Technology for an example to discuss the teaching design of such curriculums, including Big data and Financial Decision Making, Machine Learning and Intelligent Accounting, Cloud Accounting and Intelligent Financial Sharing. Also include the application of financial intelligence and big data and cultivation of intelligent tax administration ability so as to initially explore the way of combining the new generation of information technology and accounting teaching. In terms of talent demand, Lan and Chen [21] had a study on the demand of accountant talents under the environment of “Internet+” with a questionnaire. Wang and Yang [22] analyzed the change of the overall skill demands of an accounting career according to the American vocational information education network data and Chinese related recruitment data.

### 2.2. Relevant Research in Other Countries

In the past ten years, along with the fast-paced technical progress, there has been a universal resonance for the appeals of academic circle: accounting education should keep pace with the technical development [23–26] but teaching and curriculum development has not moved on at a visible speed [26]. Excel has gradually been the dominant and key technical field. By far, it has been a widely used tool with powerful functions; but there is still no similar attention for other important technologies. The existing innovations are in data analysis and many other tools (IDEA, Python, and Tableau). Therefore, there is more and more urgent demand to integrate data analysis and new technology into the curriculum of accounting [28]. Sledgianowski et al. provides a demonstration to integrate big data and information systems into teaching resources from the perspective of integration framework of accounting education ability [29]. Elsevier's affiliated accounting education journal (Journal of Accounting Education) presented a special journal for big data in 2017, which was publicized with resources to integrate big data into a class, including the free links of datasets, software tools, cases, and PPT in the class. The world's leading nongovernmental certification body for business schools and accounting programs, The Association to Advance Collegiate Schools of Business (AACSB), has recommended in the standard A7 (2013) that accounting students should take the curriculums of data creation, data sharing, data analysis, data mining, data reporting and data storage, and so on. In 2018, AACSB replaced A7 with A5: information technology skills, agility, and knowledge for accounting graduates and teachers (https://www.aacsb.edu/accreditation/standards/accounting), including five study topics and 17 specific questions: (1) impact and status of compliance implementation; (2) guide to application integration technology; (3) method of application integration technology; (4) challenges faced and resources needed; (5) which curriculums include technical skills and which software programs are used. The evolution of these standards is one of the implementation powers to push the integration of technological innovation into accounting education. Dzuranin et al. [8] suggested three possible methods to integrate technology into the cultivation and accounting talents: (1) pertinent methods (setting one key curriculum); (2) comprehensive methods (combined in multiple curriculums); (3) mixed method (being integrated to other curriculums as the main curriculum). The study result showed that most teachers supported the mixed method, and the specific implementation depended on the availability, financial support, and technical resources for teachers. Qasim (2020) built up a model to integrate data analysis on the existing accounting curriculum for undergraduates, so there was no need to provide an independent data analysis curriculum [30]. The model was designed with data analysis applications related to specific levels of learning and accounting curriculums. At the same time, many scholars would integrate one technical tool into the specific situation of the curriculum, such as using Tableau in the curriculum of audit [27]; integrating the block-chain topic into the situation and their own strengths of the curriculum of accounting for postgraduates and undergraduates [28], etc. Meanwhile, it is very necessary to have empirical study to test the impact of these new technologies on students' participation and learning and the empirical application study used to describe curriculum assignments and teachers' use of these technologies in the teaching environment (Ronald et al. 2021).

By far, current studies mainly focus on integrating technology into the concept of accounting teaching, talent cultivation scheme, curriculum integration design, and so on; while there is a lack of study on students' learning practice after integrating technology into the curriculum, especially for undergraduates. Ministry of Education of China pointed out in the “objectives and principles of building high-level undergraduate education” that we should pay attention to both “teaching well” and “learning well” when insisting on the student orientation in 2018. Hence, this project decomposes the feedback and satisfaction evaluation from students on the teaching methods and teaching contents through the text mining technology based on the data of students' learning summary text to verify the teaching effectiveness, which would provide a beneficial reference for the teaching in the future.

## 3. Research Background

### 3.1. Background of Setting up the Curriculum of “Intelligent Accounting”

By far, the traditional accounting function centered on accountancy which has been replaced by management accounting and business decision-making functions to support the decision making. The establishment of financial sharing center is a key promoter for transformation of finance. At the same time, AI technology has been accessed to accounting, audit, tax and others, and it has gradually replaced a large number of manual inputs, reviews, statistics, and other work with high repeatability. In 2020, accounting major of Beijing Union University has been approved to be top construction site in Beijing City. To cope with the challenge raised by the technical reform for the traditional cultivation of accounting talents, the team plans to set up the curriculum of intelligent accounting to integrate networking and intelligence into accounting so that students could learn the basic theory of financial sharing and get familiar with the practical operation and the whole process of financial sharing center construction. Meanwhile, they could understand real-world scenarios and actual application of RPA to master the method of primary design development. It is hoped that students could feel the necessity of transformation of corporate finance under the digital era through setting up the curriculum of intelligent accounting, and they could handle the basic business workflow with software and design a simple RPA process based on the scene when understanding the basic theories.

### 3.2. Teaching Contents and Teaching Methods of Intelligent Accounting

#### 3.2.1. Teaching Contents

In 2021, the teaching team initially sets up Intelligent Accounting for undergraduates of the whole college. The teaching contents were divided into two modules, the financial sharing center and RPA. A total of 51 students took the curriculum. There were 16 teaching weeks for the curriculum with a total of 32 learning hours. The first module was made up of enterprise digital transformation and financial digital transformation, planning and design of intelligent financial sharing center, and business process processing of intelligent financial sharing center; and the second module was composed of the development and application of artificial intelligence, which introduced a series of features and strengths of RPA and the development trend of RPA's human-computer cooperation in the future; and then the operation practice of financial RPA was displayed based on Yongyou's RPA to explain the specific application of RPA and learn how to design RPA robot.

#### 3.2.2. Teaching Methods

The teaching method is a general name of the behavior mode adopted by teachers and students in teaching activities in order to achieve the teaching purpose and teaching task requirements. The teaching methods of this curriculum consist of classroom lecturing, flipped classroom, case analysis, and simulation training. The classroom lecturing mainly includes the knowledge of the value of enterprise digital transformation, the classical model and specific path of enterprise digital transformation and financial digitalization, and the development trend of RPA's human-computer cooperation in the future. Secondly, with the full use of such teaching resources as videos and cases, it is strengthened with the preview before the class, discussion in the class, and the after-class review so as to implement the flipped classroom and rebuild the learning process. For example, the current situation of the financial control center before the establishment of a group and the current situation of a group's procurement management is displayed, and teachers are asked to discuss and sort out the pain points in the form of group; and then the discussion result of a group would be presented in the class and then teachers help students have extraction and conclusion. In addition, with the same enterprise as a case, it goes through the learning of financial sharing module to analyze the planning and design of its financial sharing center, including the strategic objectives, construction mode, construction address, and service scope; and take students' discussion in the class, such as how to choose the mode of sharing center according to the strategic objectives and how to choose the proper location according to many influencing factors of the setting of sharing center. At the same time, due to the bigger teaching difficulty of integrating intelligent technology, students should be placed in the simulated working scene through simulation training so as to learn in the financial sharing module and RPA module. It is set with expense reimbursement, purchase and sales order maintenance RPA, customer maintenance RPA, and other projects to identify different roles, and students are asked to have repeated operation in or after class; and then they should have a review and reflection after finishing the operation.

## 4. Data Available for Research and Text Mining Implementation

### 4.1. Data Sample

The data of this paper are gained from the learning summary and understanding of sophomores after having Intelligent Accounting four times in Business College. A total of 51 students took the curriculum. They majored in international business (10), finance (18), and accounting (23), including 16 boys and 36 girls. 51 students had submitted 202 texts with about 172,000 words. The main contents include students' evaluation and reflection of the learning contents and teaching methods related to the curriculum.

### 4.2. Text Mining Technology

The data source text of this research is a character string type, and the general indicators, comparative analysis, and other numerical data analysis methods are hard to be used, so the research is mainly adopted with TFIDF analysis, topic modeling, and text sentiment analysis to analyze compliant text data of the curriculum submitted by the 51 students with a visualized presentation. The problems of curriculum contents, the organization, and design of teaching would be found out by summarizing the teaching implementation effectiveness from the evaluation of students' satisfaction with the curriculum so as to propose feasible improvements.

#### 4.2.1. TFIDF Analysis

TFIDF (term frequency-inverse document frequency) is a common weighted technology used for information retrieval and data mining. It is used to evaluate the importance of a term to a document set or one of the documents in a corpus. Normally, an inverse document frequency (IDF) would be used to measure the universal importance of a term. IDF of one unique term could be gained by dividing the total number of documents by the number of documents containing the term and then taking the logarithm of the quotient. For example, the total number of terms is 100 in one paper, and there are 3 times of the term “transformation,” so the term frequency (TF) of the term “transformation” in the text is 0.03 (3/100). One method to measure the document frequency (DF) is to determine how many documents have used the term “transformation” and then divide by the total number of documents contained in the document set. Hence, if the term “transformation” shows in 1,000 documents, and the sum of the documents is 10,000,000, then the inverse document frequency would be 9.21 = (ln (10,000,000/1,000)). The score of the final TF-IDF is 0.28 = (0.03^∗^9.21).

#### 4.2.2. Topic Modeling

Topic modeling is also called topic analysis or topic extraction, which could handle a batch of unstructured and unmarked data. In the classification of robot learning, it belongs to the range of unsupervised machine learning. According to the definition in Wikipedia, the topic model means a statistical model used to find abstract topics in a series of documents in the fields of machine learning and natural language processing.

As for the use of topic modeling, it is extracted from the summary of student Xie in the first stage: “Focus on the learning atmosphere and activity degree of the class, and the lecturing style is relaxing and humorous; be able to begin from the daily life and teach with a more student-friendly method to arouse the learning interest of students effectively, so as to ensure that students could acquire something in the class. In the class, a group would be questioned randomly to catch students' attention so that everybody could focus on the classroom. Furthermore, there is a special time for the group discussion so that the members could have an exchange on their opinions, which is good for triggering brain-storming to have a profound consideration on some problems.” You would naturally know that this topic is about teaching methods after reading the text, but how do machines let readers know it? The machine would extract the terms related to teaching methods to show it, such as class, learning atmosphere, lecturing style, relaxing and humorous, so that readers could figure out the topic and the expression without reading the whole text.

#### 4.2.3. Text Sentiment Analysis

The study would extract a series of evaluation terms from data, and they would be divided into 5 degrees according to the score of text sentiment. Every 0.2 score interval is divided into one degree, 0–0.2 is worse; 0.2–0.4 is bad, 0.4–0.6 is medium, 0.6–0.8 is good, and 0.8–1.0 is excellent. In the calculation of the score of satisfaction, the median of each degree's score interval would be taken in this research, such as 0.9 for the excellent. The value of this degree can be obtained according to the proportion of the term frequency of this degree in the term frequency of the whole degree; the total score of satisfaction is the sum of the score in the five degrees.

### 4.3. Application of Text Mining Technology

This research is mixed with such text mining technologies as topic modeling, TF-IDF analysis, and text sentiment analysis, and the process is mainly included with confirming data type, confirming analysis method, preparation of compliant text, text processing, visualization presentation, result analysis, and others. The specific process is shown in Figure 1.

Firstly, because the teacher team has issued relevant requirements for the summary of each stage of the course, this study needs to initially have a primary statistic of the data quantity that meets the requirements of relevant matters, so as to eliminate the unqualified text data. Then, with the basis of the event, there is a segmentation of the text, including segmenting terms and deleting stop terms to gain the term frequency, so as to build up distributed representation conversion to structuralize data. According to the content of this study, an ontology thesaurus and synonym replacement thesaurus are built up with statistics of term frequency and the mark of the part of speech.

After finishing the data preparation, there is a topic modeling based on machine learning to extract a series of key terms to identify the analysis topics of “teaching content” and “teaching method.”

After the data preparation is completed, topic modeling is performed based on machine learning, a series of key words are extracted, and the analysis topics of “teaching content” and “teaching method” are identified. At the same time, there is a respective calculation of the score of TF and IDF for the high-frequency terms to gain the score of TF-IDF. Hence, 20 phrases with the highest scores in the teaching module of financial sharing and the RPA can be obtained based on the TF-IDF score results.

Next, the evaluation words are extracted from the established adjective thesaurus and divided into five degree intervals. Multiply the proportion of a certain degree of term frequency in the overall degree of term frequency by the median value of its degree interval, and sum up the scores of each degree interval to gain the final score of the analysis topic. In addition, the Tableau tool is used to have the biterm analysis on the high-frequency terms of the analysis topic, “teaching contents” and “teaching methods” and the degree terms of “excellent” and “bad”; and then there is an interpretation on the terms with a high frequency of occurrence. At the same time, there is a comparison of the score of curriculum module of financial sharing center and RPA to highlight students' satisfaction of the teaching contents and the teaching methods.

## 5. Analysis of Students' Satisfaction

### 5.1. Confirmation of the Degree Grade of Teaching Satisfaction

Through retrieving the data of students' summary text, there is analysis on the sentiment of the degree, and the adjective terms are transformed to be the measurable and specific measurement standard to have the analysis of satisfaction evaluation on the teaching contents and the teaching methods. The classification of degree terms is shown in Table 1.

### 5.2. Analysis of Satisfaction of Teaching Contents

The summary text of the module of financial sharing center is made as the statistical sample to have the biterm frequency analysis of “teaching contents” and degree term. It can be seen from Table 2 that the term frequency of the co-occurrence of the “excellent” with teaching contents is the highest, which accounts for about 42%; while the term frequency of that with “good” accounts for 19% approximately; the proportion of the two terms is 61%. The sum of the score of teaching contents is 0.653, within the interval of 0.6–0.8, which indicates that most of the students have a higher satisfaction on the teaching contents of the financial sharing center.

To further refine the teaching contents, there is a specific analysis of the two-degree terms with the highest proportion, “excellent” and “bad.” This study has a biterm analysis on the degree terms of “excellent” and “teaching contents.” It could be easily found that (seen in Figure 2) such terms as “learning,” “accounting,” “Internet,” “financial sharing center,” and “analysis” in the teaching contents have higher term frequency, which partly reflects that most of the students have a high satisfaction on the teaching contents involved in the financial sharing center and the accounting knowledge of the Internet.

For the biterm analysis of “bad” and the “teaching contents,” as shown in Figure 3, the terms with higher frequency are “Internet,” “curriculum,” “learning,” “accounting,” etc. Obviously, some students may have a negative tendency for the teaching contents of intelligent accounting. These students have been less exposed to content. The contents of curriculum are innovative, but there are such terms to show the laborious learning as “cannot keep up,” “absent-minded,” “esoteric,” and “slow it down.” However, they are not very resistant to the teaching content. They will tend to keep studying, but they are unsatisfied with the arrangement of learning hours. In the follow-up lectures, teachers could try to change other organizational methods of teaching so that the students with poor basis could keep pace with the learning.

Then, the paper takes the summary text of the module of the RPA financial robot as a statistics sample to have a term frequency analysis of “teaching contents” and degree terms. As shown in Table 3, the term frequency of the co-occurrence of “excellent” with teaching contents is the highest, which accounts for about 43%; while the term frequency of that with “good” accounts for 7% approximately; the proportion of the two terms is 50%. The sum of the score of teaching contents is 0.621, within the interval of 0.6–0.8, which indicates that most of the students have a higher satisfaction on the teaching contents of RPA financial robot.

To further refine the teaching contents, there is a specific analysis of the two-degree terms with the highest proportion, “excellent” and “bad.” The study has a biterm analysis on the degree terms of “excellent” and “teaching contents.” It could be easily found that (seen in Figure 4) such terms as “RPA,” “robot,” “work,” “software,” and “operation” in the teaching contents have higher term frequency, which partly reflects that most of the students have a high satisfaction on the teaching contents involved in the RPA robot, system operation, and software.

While through the biterm analysis of “bad” and “teaching contents” (shown as Figure 5), it is found that the terms with higher frequency are “RPA,” “robot,” “learning,” “software,” etc., which could be seen that some students may have a certain negative tendency on the teaching contents of RPA module. These students have access to less content. The contents of the curriculum are innovative, but there are terms to show that these students are subjectively inadaptable to the teaching contents and the knowledge is too recondite to understand, such as “cannot keep up,” “absent-minded,” “hard to begin,” “totally at loss,” and “confusing.”

### 5.3. Analysis of the Satisfaction of Teaching Methods

According to the classification of teaching methods in the curriculum combined with the description and preferences of students' summary texts, this study sorts out the relevant descriptions of students on the teaching methods to form a teaching method thesaurus for the curriculum (shown in Table 4).

Then, this research takes the summary text of the four stages as a statistics sample to have a term frequency analysis of “teaching methods” and degree terms (shown in Table 5). The term frequency of the co-occurrence of “excellent” with teaching methods is the highest, which accounts for about 44%; while the term frequency of that with “good” accounts for 16% approximately; the proportion of the two terms is 60%. And the sum of the score of teaching methods is 0.649, within the interval of 0.6–0.8, which indicates that most of the students have a higher satisfaction on the teaching methods adopted by the curriculum.

To further analyze the teaching methods that are favored or hated by students, this research divides the methods into teaching method, flipped classroom, simulation training, and case analysis according to the degree terms subdivided depending on different teaching methods. The analysis of satisfaction evaluation for different teaching methods is shown in Table 6.

#### 5.3.1. Classroom Lecturing

This study divides the classroom lecturing into four parts, including theoretical explanation, language, thinking, and attitude; and there is a biterm frequency analysis of the different parts and the degree terms, as shown in Table 7.

It could be seen that both theoretical explanation and attitude get the highest score with the highest satisfaction; while there are fewer evaluation terms on language and thinking, so there is a gap with the theoretical explanation in view of satisfaction. Hence, by retrieving the data of this part, it could be seen that there are “unfamiliar”, “short time”, “cannot keep up with the thinking” and other terms, which shows that students are unsatisfied with the time length and the speed of teaching. Hence, in subsequent curriculum, teachers could provide lecture notes for students to ask them to have a preview to improve the participation, or teachers could reduce the teaching speed in the class so that students could have sufficient time to take in the knowledge to lay a solid foundation for their learning in the follow-up curriculums.

#### 5.3.2. Flipped Classroom

This study divides the flipped classroom into group discussion, cooperation, interaction mode, and self-learning these four parts, and there is a biterm frequency analysis of the different parts and the degree terms.

As seen from Table 8, the score of self-learning is the highest, 0.8, so students have the highest satisfaction on this part. The general evaluation terms of self-learning are less, and most of these samples are positive, so the evaluation of self-learning is the highest. The scores in group discussion, cooperation, and interaction mode are higher with the better satisfaction, but there are term frequencies of “bad” and “worse.” Hence, by retrieving the data, it could be seen that there are terms of “unfamiliar group members” and “personal opinions,” which means that students are unsatisfied with the grouping arrangement. In the teaching improvement of the curriculum, teachers could consider allowing students to form groups by themselves to enhance the familiarity and give them enough time to take the group activity to strengthen their ability of self-learning.

#### 5.3.3. Simulation Training

The study divides the simulation training into practice, knowledge application, simulation practice, Yonyou, Seentao Cloud these six parts, and there is a biterm frequency analysis of the different parts and the degree terms.

As seen from Table 9, the scores of Seentao Cloud and Yonyou are the highest, 0.7 and 0.717, respectively, which means that students have the highest satisfaction on these two parts. However, the general evaluation terms of these parts are less, and most of these samples are positive, so the evaluations are the highest. By retrieving the data, it could be seen that there are terms of “unfamiliar Seentao Cloud platform” and “do not know how to operate the platform,” which means that teaching of the new platform is a little hard work and maladjustment for a small number of students. However, the problem would be properly improved along with the further undertaking of the curriculum.

At the same time, it could be seen from observing the data of other parts that the score of other parts is higher with higher satisfaction, but there is such frequency terms as “bad” and “worse.” Hence, after retrieving the data, it could be found that there are terms in the part of the operation practice in laboratory, including “slow network speed,” “slow it down,” “computer configuration,” and “old and backward hardware,” which indicates that students have no subjective resistance on the teaching methods but the restriction on objective condition. In view of the part of homework, there are such terms as “less homework,” “have no idea to begin the homework,” and “give more time”, which means that the distribution of practice homework is a little hard work for a small number of students.

#### 5.3.4. Case Analysis

As shown in Table 10, students have a better acceptance of the teaching methods of case analysis. By retrieving the data of this part, it could be gained with such terms as “Hongtu Group,” “World Coffee,” “Decathlon,” and “Xiangyue Sports Group,” which shows that students are impressed with these cases, and their ability to apply knowledge has been improved through case analysis. However, a small number of students are unsatisfied with it since there are such terms as “increase case,” “case in life,” and “data of actual case”, which shows that students have a good adjustment to the part of case analysis and raises the higher requirement accordingly.

## 6. Discussion and Conclusion

On the whole, the students are satisfied with the teaching contents and teaching methods of Intelligent Accounting. This study observes the scores comparison of the teaching contents and teaching methods in the two curriculum modules with propensity scores. The proportion of all degree terms in teaching contents and teaching methods of the two curriculum modules could be concluded from Tables 2, 3, and 5 and correspondent methods, and then multiply the proportion by the median of each score interval to obtain the score of each item, as shown in Table 11.

Since the highest score adopted by the study is within the interval of 0.8–1 with the median of 0.9 and the minimum of 0.1, the satisfaction scores of all items are higher. As seen from the score comparison, both the teaching contents and teaching methods of the RRA curriculum module are worse than those of the curriculum module of the financial sharing center. On the one hand, along with the proceeding of curriculum, students' attention to the curriculum may decline; on the other hand, partial students have difficulty in learning of the curriculum module of RPA, and they suffer from such terms as “cannot keep up” and “hard to begin.” The reasons for the problem are the following. One is that the contents of RPA need the actual drill, and the new learners (most of them have not learned computer science) need teachers to slow it down to have a specific explanation. Hence, teachers could try to provide lecture notes and ask them to have a preview to improve the participation in the class or properly reduce the teaching speed; or teachers could try some new teaching ways, such as having a drill of the process of practical operation with training aid, asking students to operate when thinking to deepen the impression. The other reason is the hardware issue in the laboratory. The operation software of RPA needs a certain hardware basis, so the students' satisfaction would be reduced when the RPA robot running is unstable due to the slow network speed and low computer configuration in the machine room.

In the future lecturing, teachers could try to improve teaching satisfaction from the two perspectives. Firstly, for the RPA module, teachers could upgrade the hardware in the laboratory or consider asking students to take their own computer and ask them to make configurations in advance. Secondly, in view of some students with the term “cannot keep up,” teachers could designate some simple practical operation as after-class practice in advance. On the other hand, the students who have been proficient in the training should be cultivated in the group to work with teachers in leading others. In future teachings, teachers should keep paying more attention to students' understanding and acceptance and continuously listen to their demands. Teachers should value not only the “teaching” but also the “learning” to keep upgrading the teaching satisfaction in the review and reflection of teaching.

Consequential curriculum innovation appears for an intimidating and significant challenge that often falls short of a priori objectives for the programs. We find preliminary evidence that suggests further improvement of the teaching contents and optimization of the teaching design to effectively improve the curriculum quality so as to achieve enhancement of students' satisfaction. Additionally, this research considers the impact of technology evolution specifically within undergraduate curriculum required of all business majors to sufficiently adapt to the changing role of the occupation. We believe that this research is an important initial step towards revisiting the business curriculum and helping future research explore additional opportunities across business program.

## 7. Limitations and Future Research

Our study is subjected to several limitations that are common to research design. Foremost, the population of students all being mates of the same college and their response may create potential for biased results, although we have no reason to believe that any specific bias exists. Secondly, there is a general lack of control over who responds to a survey [29]. In addition, survey research can capture attitudes and opinions at a point in time, which provides the evidence of correlation, but cannot determine cause and effect relationships. Many possible future research opportunities exist. Comparisons might be made among potential students from various colleges and different programmes. A more in-depth analysis is warranted from the present study's results.

## Figures and Tables

**Figure 1:** Process of text mining.

**Figure 2:** Biterm analysis of teaching contents and the degree term, “excellent.” Note: term A refers to teaching contents and term B indicates the term of excellent.

**Figure 3:** The biterm analysis of teaching contents and the degree term, “bad.” Note: term A refers to teaching contents and term B indicates the term of bad.

**Figure 4:** Biterm analysis of teaching contents and the degree term, “excellent.” Note: term A refers to teaching contents and term B indicates the term of excellent.

**Figure 5:** The biterm analysis of teaching contents and the degree term, “bad.” Note: term A refers to teaching contents and term B indicates the term of bad.

**Table 1:** Induction of degree terms.

Worse (0∼0.2)	Bad (0.2∼0.4)	Medium (0.4∼0.6)	Good (0.6∼0.8)	Excellent (0.8∼1.0)	
Completely confusing	Cannot keep up	A little bit vague	Have gained something	Easily approachable	Happy learning
Cannot understand it	Slow down a little	A little bit too fast	Apt to understand	Vivid language	Very novel
Solo lecture	A little slower	Not bad	Clear and understandable	Well organized	Draw upon all useful opinions
Too blunt	Slow it down	Okay	Easy to understand	Serious and responsible	More acceptable
Very difficult	Do not totally understand it	Interesting	Relaxing and humorous	Stimulate creative potential	Very diversified
So difficult	Do not totally get it	Serious	Better to receive	Passion	Very interesting
Hard to understand	Not too high	Not too much different	Stronger	Vivid	Very reasonable
Totally at loss	Do not understand it	Not boring	Practice coordination and cooperation	Young and energetic	High comment
Hard to identify	Do not get it	Moderate	Innovative	Like it so much	Very flexible
Hard to begin	Mess around		Humorous and funny	Very clear	Very suitable
	Bad discipline		Meticulous	So considerate	Highly efficient
	Not too good		Sincere and meticulous	Learn a lot	Very interesting
	A little bit difficult		Apt to absorb	Well promoted	Like it so much
	Embarrassing		Not boring	Serious explanation	Very good impressive
	Stiff		Exercise	Learn so much	
	Relatively conventional		Coordination and cooperation		

**Table 2:** Statistics of term frequency of degree terms of teaching contents.

Degree term	Term frequency	Proportion (%)	Score
Excellent	18	42	16.2
Good	8	19	5.6
Medium	7	16	3.5
Bad	9	21	2.7
Worse	1	2	0.1
Sum	43		0.653

**Table 3:** Statistics of term frequency of degree terms of teaching contents.

Degree term	Term frequency	Proportion (%)	Score
Excellent	24	43	21.6
Good	4	7	2.8
Medium	12	21	6
Bad	14	25	4.2
Worse	2	4	0.2
Sum	56		0.621

**Table 4:** Description thesaurus of teaching methods for the curriculum.

Classroom lecturing	Flipped classroom	Simulation training	Case analysis
Explain carefully	Group discussion	Practice	Case
Narrate	Cooperative analysis	Homework	Classic case
Very clear	Cooperation and coordination	Finish homework	Real case
Declare	Interaction	Task work	Relevant case
Lecture	Group setting	Learning task	Case analysis
Easy to understand	Group form	Yongyou	Classroom case
Serious teaching	Assemble group	Ability of practical operation	Case discussion
Clear and understandable	Select group	Practical operation	Hong Tu
Well organized	Group cooperation	Seentao cloud	Decathlon
Theoretical explanation	Group collaboration	Writing	Lining
Clear thinking	Divide into groups	Operation	Hongtu
Explain clearly	Self-learning	Sand table	Bensteel
Theoretical explanation	Exploration	Do	China communications construction

**Table 5:** Statistics of term frequency of degree terms of teaching methods.

Degree term	Term frequency	Proportion (%)	Score
Excellent	33	44	29.7
Good	12	16	8.4
Medium	14	19	7
Bad	10	13	3
Worse	6	8	0.6
Sum	75		0.649

**Table 6:** Classification of teaching methods.

Classroom lecturing	Flipped classroom	Simulation training	Case analysis
Theoretical explanation	Group discussion Cooperation Interaction Self-learning Divide into groups	Practice Knowledge application Simulation Finish homework Yonyou Seentao cloud	Hong Tu
Attitude			Decathlon
Language			Xiangyue sports group
Thinking			World coffee

**Table 7:** Analysis of term frequency of classroom lecturing.

Classroom lecturing	Excellent	Good	Medium	Bad	Worse	Score
Theoretical explanation	28	22	14	8	1	0.686
Attitude	1	2	0	0	0	0.767
Language	7	5	2	3	1	0.656
Thinking	1	3	0	2	0	0.600
Sum	37	32	16	13	**2**	**0.667**

**Table 8:** Analysis of term frequency of flipped classroom.

Flipped classroom	Excellent	Medium	Bad	Worse	Score
Group discussion	13	6	5	1	0.666
Cooperation	6	4	3	0	0.662
Interaction mode	16	6	3	2	0.689
Self-learning	1	0	0	0	0.800
Sum	**36**	**16**	**11**	**3**	**0.677**

**Table 9:** Analysis of term frequency of simulation training.

Simulation training	Excellent	Good	Medium	Bad	Worse	Score
Practice	33	22	15	7	5	0.673
Knowledge application	17	17	9	11	2	0.629
Simulation practice	10	6	6	4	3	0.610
Homework	17	12	14	5	3	0.637
Yonyou	9	8	5	1	0	0.717
Seentao cloud	2	0	0	1	0	0.700
Sum	88	65	49	29	13	**0.647**

**Table 10:** Analysis of term frequency of case analysis.

Case analysis	Excellent	Good	Medium	Bad	Worse	Score
Case	11	7	7	2	0	0.700

**Table 11:** Comparison of curriculum modules of financial sharing center module and RPA curriculum module.

Curriculum module	Financial sharing center		RPA	
Item	Teaching contents	Teaching methods	Teaching contents	Teaching methods
Score	0.653	0.696	0.621	0.615

## Data Availability

All the data used to support the findings of this study are available from the corresponding author upon request.
